This article has been retracted.

# Effect of Vitapex Combined with AH-Plus Paste on Inflammation in Middle-Aged and Elderly Patients with Periodontal-Endodontic Disease

**DOI:** 10.1155/2022/7540961

**Published:** 2022-07-01

**Authors:** Rong Hu, Fulan Zhang, Xiangyu Guo, Youren Jing, Xiaowan Lin, Liping Tian

**Affiliations:** ^1^Eastern Clinic, West China Hospital of Stomatology Sichuan University, 610051, China; ^2^Wuhan, Hankou Hospital Department of Stomatology, 430000, China; ^3^Wuhan Wuchang Hospital, Wuchang Hospital Affiliated to Wuhan University of Science and Technology, 430063, China

## Abstract

**Aims:**

To investigate the effect of Vitapex combined with AH-plus paste on inflammation in middle-aged and elderly patients with periodontal-endodontic disease.

**Materials and Methods:**

A total of 80 teeth of middle-aged and elderly patients with the periodontal-endodontic disease who were treated in our hospital from June 2020 to June 2021 were selected as the research objects and were divided into comparison group and treatment group with 40 teeth each according to different treatment methods. Among them, the comparison group was filled with zinc oxide clove oil paste gutta-percha, and the treatment group was filled with Vitapex combined with AH-plus paste. The changes in apical cross-section sealing performance, periodontal pocket depth (PD), and gingival index (GI) of the two groups before treatment and after 6 months of follow-up were observed and compared, and X-ray analysis was performed.

**Results:**

There was no significant difference in the level of periodontal indexes and serum inflammatory indexes between the two groups before treatment (*P* > 0.05). After treatment, the levels of PD, BI, PLI, and GI in the two groups were significantly lower than before treatment (*P* < 0.05). The differences in IL-6, IL-10, TNF-*α*, and IL-1*β* after treatment were significant (*P* < 0.05). There was no significant difference in the root canal area data of each cross-section between the two groups when the root canal was filled with root filling paste at different positions from the apex (*P* > 0.05). After root canal filling with root canal paste, the cross-sectional area from different parts of the root canal in the treatment group was significantly smaller than comparison group (*P* < 0.05). After 6 months of treatment, it was found that CEJ-BD and CEJ-AC in the treatment group were significantly lower than those in the comparison group (*P* < 0.05).

**Conclusion:**

Vitapex combined with AH-plus paste filling can effectively treat middle-aged and elderly periodontal-endodontic disease, which provides a certain reference for the clinical treatment of middle-aged and elderly periodontal-endodontic disease.

## 1. Introduction

Gum-related endodontic disease refers to the damage to body parts of the gum-related tissue and pulp tissue of the same tooth, often showing dual signs of gum swelling and pulpitis, a common and complex oral disease in medicine-based [1]. Both the pulp and gum-related tissues develop in mesodermal tissue so that there is a complex relationship between the two in structure and function, overlying structures such as dentinal tubules protect diffusion [2]. Thus, it can also affect other tissues when disease-related changes occur in tissues, leading to corresponding signs of disease and signs in tissues. [3]. Although the disease-causing factors and disease-related changes of gum swelling and pulpitis are not the same, most people think that these two sicknesses are mainly mixed bacterial infections [3]. Patients with the gum-related-endodontic disease are in poor general condition and compared to other things extreme disease at the time of discussion with other people because of the living together of signs of endodontic disease and gum-related disease [4].

Through the related to the tip foramen, the lateral and added or extra someone or something that helps root narrow, human-made waterways and dentinal tubules communicate with each other related to body structure. The gum-related and pulp tissues communicate with each other, and there are mixed infections ruled by not needing oxygen bacteria in the gum-related pockets and the infected pulp [5]. Perfect root narrow, human-made waterway treatment plays an important role in gum-related endodontic disease. If the endodontic treatment is not complete, it will seriously affect the treatment effect. Different root filling pastes have different medicine-based effects. Vitapex combined with AH-plus paste is used, to determine the worth, amount, or quality of the medicine-based healing effect of gum-related pulp tissue after a root filling. Vitapex paste is a pressurized injectable root narrow, human-made waterway filling material whose main parts are silvery important nutrient hydroxide, iodoform, and silicone oil [6]. AH-plus is a sticky, plastic-like substance that usually comes from trees root filling paste with high X-ray resistance and low ability to be dissolved in something. Its main parts are an epoxy sticky, plastic-like substance that usually comes from trees, important nutrient tungstate, zirconia, silica, amine, and excipients. It is based on epoxide amine sticky, a plastic-like substance that usually comes from trees chemically and is easy to mix. It has no obvious shrinkage after an act of turning into a solid, can reduce a lot of the pain response after root narrow, human-made waterway, effectively controls periapical swelling, and has good biocompatibility [7]. Based on this, we made some events where things have explored the effect of Vitapex combined with AH-plus paste on swelling in middle-allowed to get old and old patients with the gum-related endodontic disease.

## 2. Material and Methods

### 2.1. Research Object

Before participating in this study, patients were fully introduced to the content of the experiment, the process, the associated risks, and possible adverse reactions. After the patient agrees, they signed an informed consent form, and the patients were informed of the final test results. Eighty teeth of middle-aged and elderly patients with periodontal-endodontic disease who were treated in our hospital from January 2021 to December 2021 were selected as the research objects. The materials used are as follows: Vitapex paste (Morita Co., Ltd., Japan); AH-plus paste (Dentsply, Germany); ultrasonic scaler (EMS, Switzerland); Gracey subgingival scaler (Hu-Friedy, USA); Root ZX root canal measuring instrument (Morita, Japan); and ProTaper machine root canal instrument (Dentsply/Maillefer, Switzerland). The general data of the patients in the two groups had no effect on this trial (Table 1).

### 2.2. Patient Eligibility Criteria

Inclusion criteria are as follows: (i) All patients in this study met the diagnostic criteria for middle-aged and elderly periodontal-endodontic disease in the “Standardized Diagnosis and Treatment of Periodontal-Endodontic Lesions” [8]. Bite pain or weakness, gingival pus, redness and swelling, and lower dental calculus I-III degree are shown; X-ray films show some teeth caries, crown loosening, low-density images in the apical area of teeth, crest, or alveolar root apex. There are different degrees of resorption at the bifurcation, accompanied by a history of spontaneous pain; (ii) there is loss of attachment, true periodontal pockets, and degree of tooth mobility, the crown of the affected tooth is intact, there are no caries, and there are symptoms of irreversible pulpitis or pulp vitality test, negative; (iii) X-ray films showed that the alveolar crest or root bifurcation had different degrees of absorption, and there were different degrees of low-density shadows around the root apex.

Exclusion criteria are as follows: (i) there is calcification or mutation of the root canal, it is difficult to use root canal treatment, and extraction or surgery is used; (ii) patients with severely impaired immune function, accompanied by renal function damage, severe thyroid disease, accompanied by major diseases and other typical cachexia; and (iii) patients who have systemic diseases, have received periodontal treatment in the past 12 months, have a history of drug allergy, and are pregnant or lactating women.

## 3. Intervention Methods

Both groups went through basic gum-related treatment, including supragingival scaling, subgingival scaling with ultrasonic cleaning, and Gracey scaler to complete subgingival scaling, root planing, occlusal change to make better/related to changing something, and improved oral keeping yourself/something clean guidance. The comparison group was filled with zinc oxide clove oil paste gutta-percha. That is, the root narrow, human-made waterway was filled with zinc oxide clove oil paste lateral pressure filling method after sealing Ca(OH)_2_ for 1 week. The treatment group was used with Vitapex combined with AH-plus paste filling, namely Vitapex paste plus gutta-percha tip filling. Insert the Vitapex paste syringe into the root narrow, human-made waterway, slowly inject the paste, and slowly withdraw along one side of the root narrow, human-made waterway wall while injecting the paste. When the yellow paste overflows from the root narrow, human-made waterway opening, remove the syringe. Apply a small amount of Vitapex paste evenly to the tip of the main gutta-percha tip, slowly insert it into the root narrow, human-made waterway according to the operating length, pressurize with a not extreme/medium-level lateral presser, keep it for the 30 s, then fill it with the secondary tip, apply Vitapex to the tip before filling Paste, pressurize with a side presser until the side presser is inserted into the root narrow, human-made waterway 3 mm away from the root narrow, human-made waterway opening, and finally cut off the excess gutta-percha tip with a thermal tool or object used to do work or measure something. Review after 1 month, remove the paste in the root narrow, human-made waterway, replace the AH-plus paste, bring the prepared AH-plus paste with a 30#K file to the operating length, and then rotate the K file when a wheel turns, so the top moves to the left. Withdraw the root narrow, human-made waterway, and do this over and over again so that the whole root narrow, human-made waterway is filled with AH-Plus paste. Apply a small amount of paste to the tip of the main gutta-percha tip. All experimental medical examples after the above operations were sealed with zinc phosphate cement for a short time, and X-ray films of all medical samples/examples were taken in each direction to check the tightness of root filling. To remove the far apart from others tooth with incomplete root narrow, human-made waterway, the above operations should be done by the same person who works to find information.

## 4. Observation Indicators

Periodontal indexes are as follows: periodontal pocket depth (PD), bleeding index (BI), plaque index (PLI), and gingival index (GI) before and after treatment in the two groups. Serum index is as follows: For the patients included in the trial, 1 ml of whole blood (using a sterile tube) was collected before treatment (on the day of participating in the trial) and after treatment, centrifuged at 1000 × g for 20 minutes (4°C) overnight, taken, subpackaged supernatant, and placed in a -80°C refrigerator for detection of IL-6, TNF-*α*, IL-10, and IL-1*β*. The periodontal probing depth (PD), bleeding on probing index (BOP), and gingival index (GI) were measured and recorded on the day of baseline and 6 months later, and the preoperative and postoperative X-ray films were recorded by the parallel projection method, Dimaxis Pro4. The 0.2 software measured the distance from the cementoenamel junction to the bottom of the bone defect (CEJ-BD) and the alveolar ridge top (CEJAC) in the X-ray films. All the root canal cross-section specimens were scanned by scanning electron microscope and input into the computer through the scanner to measure the void area on each cross-section and the total area of the root canal in the cross-section, and the root canal in each cross-section of each specimen in the two groups was calculated. The area and the percentage of void area therein (PV) were recorded. Percentage of void area = (area of void on this slice section/root canal area of this slice section) × 100%.

## 5. Statistical Analysis

All the statistical data in this study were tested by the Shapiro-Wilk method. Mean ± standard deviation (*x̅*±*s*) was used to describe the measurement data conforming to the normal distribution. The between-groups or the independent-sample or paired-sample *t*-test was implemented within the group. Count data is described as integers or percentages (%), and the *χ*^2^ test is used between or within groups. *M* (QR) describes data that do not conform to the normal distribution and uses the Mann-Whitney test, which is tested at a level of *α* = 0.05.

## 6. Results

### 6.1. General Data

The difference in general clinical data (such as the gender, average age, disease course, degree of tooth loosening, etc.) of the patient's teeth showed that there was no significant difference in general clinical data between the two groups (*P* > 0.05), and the two groups were comparable (see Table 1).

### 6.2. Periodontal Index

Before treatment, there was no significant difference in the periodontal index levels between the V-AH and the comparison groups (*P* > 0.05). After treatment, the PD, BI, PLI, and GI levels in the two groups were lower than before, and the treatment group was significantly lower than the comparison group (*P* < 0.05) (see Figure 1).

### 6.3. Serum Inflammatory Markers

There was no significant difference in serum inflammatory indexes between the two groups before treatment (*P* > 0.05), but there were significant differences in IL-6, IL-10, TNF-*α*, and IL-1*β* between the two groups after treatment. It was significantly better than the comparison group (*P* < 0.05) (see Figure 2).

### 6.4. Comparison of Sealing Performance of Root Apex Cross-Section

The follow-up after 6 months of treatment showed no significant difference in the root canal area data between the two groups at different parts of the root canal from the root apex (*P* > 0.05). After root canal filling with root filling paste, the cross-sectional area of different parts from the root apex in the treatment group was significantly smaller than that in the comparison group (*P* < 0.05) (see Figures 3 and 4).

### 6.5. Periodontal Bone Defect and Alveolar Crest Bone Mass Change

After 6 months of treatment, follow-up showed that the CEJ-BD and CEJ-AC of the treatment group were significantly lower than those of the comparison group (*P* < 0.05) (see Figure 5).

## 7. Discussion

The medicine-based number of times something happens of gum-related endodontic disease is high. Gum-related disease and endodontic disease can interact to a certain extent so that a tooth suffers double damage [9]. In teeth with a gum-related endodontic disease, the degree of pulpal disease directly affects the degree of gum-related disease, so the degree of perfection of root narrow, human-made waterway treatment directly affects the healing of gum-related disease [10]. Root narrow, human-made waterway therapy is now a widely used method for treating periapical damage to body parts and pulpitis. In this process, root narrow, human-made waterway filling is a very critical step, and it is necessary to make sure that the filling material puts into action its disinfection effect slowly and lastingly while blocking to eliminate the leftover infection factors in the root narrow, human-made waterway and help increase/show in a good way root highest point healing [11]. AH-Plus paste is one of epoxy sticky, plastic-like substances that usually come from trees root filling pastes. Its composition is bisphenol epoxy sticky, plastic-like substance that usually comes from trees, which has strong stickiness/scar to gutta-percha tip and root narrow, human-made waterway wall. The total space occupied by something turned into a solid paste is basically the same. There is no change in the above good firm and steady nature/lasting strength, no large thermal act of something getting bigger, wider, etc. and cold contraction, good related to space or existing in space firm and steady, lasting nature, good smoothness, and can go along with the shape of the root narrow, human-made waterway after forming, the formaldehyde content in the paste is high, Swelling of infected root narrow, human-made waterways can be effectively controlled [12]. The main pieces of Vitapex paste are silvery important nutrient hydroxide, iodoform, and polysiloxane oil. It is a new type of root narrow, human-made waterway filler [13]. Among them, polysiloxane oil is a high-grade greasing oil, which can improve the smoothness and ability to take up understandability of the paste; iodoform can play the role of germ-killing, disinfecting, reducing exudation, and deodorization and can help increase/show in a good way the mental concentration up of a liquid of insulting damage to body parts and cause gum-related tissue, related to remaking generating electricity repair [14].

In this study, the levels of PD, BI, PLI, and GI in the two groups of patients after treatment were lower than those before treatment, and the treatment group was lower than the comparison group, indicating that Vitapex combined with AH-plus paste filling can be effective in the treatment of middle-aged and elderly periodontal-endodontic disease better. The reasons are as follows. Root canal filling is an important method for the clinical treatment of periodontal-endodontic disease, and the choice of filling material has a great influence on the treatment effect [15]. As a new type of root canal filling material, Vitapex paste is mainly composed of calcium hydroxide, polysiloxane oil, and iodoform. Calcium hydroxide has a good killing effect on anaerobic bacteria and can stimulate calcified tissue formation [16]. It can promote the formation of the root apex; iodoform can play the role of antiseptic, bactericidal, and astringent and effectively promote the absorption of inflammatory lesions [17]. AH-Plus paste is one of the epoxy resin root filling pastes. Its composition is bisphenol epoxy resin, which strongly attaches to the gutta-percha tip and root canal wall. The volume of the solidified paste is basically the same. There is no change in the above, the stability is good, and there is no large thermal expansion and contraction [18]. AH-Plus paste has good spatial stability and fluidity and can conform to the shape of the root canal after forming. The formaldehyde content of the paste is high, which can effectively control the inflammation of the infected root canal [19–22].

In this study, the cross-sectional area of the root canal from the root canal filled with root filling paste in the treatment group was significantly smaller than that in the comparison group, and the CEJ-BD and CEJ-AC in the treatment group were significantly lower than those in the comparison group, indicating that Vitapex combined with AH-plus paste. The density of the filling is better, for the root canal area of each cross-section at different parts of the root canal from the root apex and the different parts from the root apex. The results of this experiment show that Vitapex paste has the following advantages: it can promote tissue ossification and calcification; the paste composition is stable and has good fluidity; macrophages can phagocytose it and has the effect of inducing root tip tissue development and effective prevention of secondary root resorption [23–25]. However, it also has certain defects, resulting in its poor compactness. After the tissue absorbs the paste filling, it will solidify and shrink and release iodine, resulting in microleakage. The paste decreases when an infection occurs, resulting in a reduced seal of the root tip after the filling period [26]. Some data show that AH-Plus paste belongs to the epoxy resin matrix, which has good fluidity, can be dissolved and absorbed in tissues, has a short setting time, and has excellent permeability. The AH-Plus paste was accompanied by a little volume expansion during its gradual solidification, with a proportion of 0.9%, and less microleakage occurred after Vitapex was combined with AH-plus paste [27].

In this study, the differences in IL-6, IL-10, TNF-*α*, and IL-1*β* after treatment were significant, and the treatment group was better than the comparison group, indicating that the addition and subtraction of periodontal-endodontic disease had obvious effects and could reduce the level of serum inflammatory indexes. IL-6 can induce inflammatory responses, and its products come from various sources. A large number of experimental data show that IL-6 is an important proinflammatory factor involved in various inflammatory responses and diseases in the human body [28]. The expression level of IL-6 in the human body will decrease to a certain extent and gradually approach a healthy level. This is because IL-6 can activate T lymphocytes, induce the differentiation of B lymphocytes, and finally secrete immunoglobulin, thus playing a role. IL-10 is also an important immune system regulator in the human body. It plays an important role in the pathogenesis of various diseases and is currently recognized by the medical community as an immunosuppressive factor [29–32]. TNF-*α* is a multifunctional inflammatory cytokine, mainly produced by eosinophils and monocytes, and has anti-infective effects. TNF-*α* can stimulate the proliferation of B cells, promote the secretion of Ig, and promote the release of inflammatory factors. TNF-*α* can affect the body's anti-infection ability, and the more severe the viral infection or bacterial infection, the higher the level of TNF-*α* [33, 34].

## 8. Conclusion

To sum up, Vitapex combined with AH-plus paste filling can be effective in the treatment of middle-allowed to get an old and old gum-related endodontic diseases. For the root narrow, the human-made waterway area of each thin slice can be looked at different parts from the root narrow, human-made waterway and the different parts from the root's highest point. The density of Vitapex combined with AH-plus paste filling is good, which provides a certain reference for the medicine-based treatment of middle-allowed to get old and old gum-related endodontic diseases.

## Figures and Tables

**Figure 1:** Comparison of periodontal indicators. (a) PD levels; (b) BI level; (c) PLI level; (d) GI levels. Values were expressed as mean ± standard deviation according to the test criterion of *α* = 0.05 and analyzed by independent-sample *t* − test.

**Figure 2:** Comparison of serum inflammatory markers. (a) IL-6 levels; (b) IL-10 level; (c) TNF-*α* level; and (d) IL-1*β* levels. Values were expressed as mean ± standard deviation according to the test criterion of *α* = 0.05 and analyzed by independent-sample *t*-test.

**Figure 3:** Comparison of root canal area in cross-section. According to the test standard of *α* = 0.05, the value was expressed as the mean ± standard deviation and passed through independent-sample *t*-test for analysis.

**Figure 4:** Comparison of percentage of void area. According to the test standard of *α* = 0.05, the value was expressed as the mean ± standard deviation and passed through independent-sample *t*-test for analysis.

**Figure 5:** Comparison of sealing performance of root apex cross-section. (a) CEJ-BD; (b) CEJ-AC. According to the test standard of *α* = 0.05, the values were expressed as the mean ± standard deviation and analyzed by independent-sample *t*-test.

**Table 1:** Comparison of general data (*n*, *x̅*±*s*).

Group	Gender (men/women)	Average age (age)	Course of disease (year)	Degree of tooth loosening	
				I	II
Comparison group (40)	18/22	53.50 ± 1.32	5.6 (3.7~7.9)	12	28
Treatment group (40)	17/23	52.69 ± 3.66	5.5 (3.1~7.7)	16	24
*χ* ^2^/*t*	0.051	1.317	0.040	0.879	
*P*	0.822	0.129	0.965	0.348	

## Data Availability

No data were used to support this study.
